RETRACTED

# Effects of CREB1 gene silencing on cognitive dysfunction by mediating PKA-CREB signaling pathway in mice with vascular dementia

**DOI:** 10.1186/s10020-018-0020-y

**Published:** 2018-05-03

**Authors:** Xin-Rui Han, Xin Wen, Yong-Jian Wang, Shan Wang, Min Shen, Zi-Feng Zhang, Shao-Hua Fan, Qun Shan, Liang Wang, Meng-Qiu Li, Bin Hu, Chun-Hui Sun, Dong-Mei Wu, Jun Lu, Yuan-Lin Zheng

**Affiliations:** 1 Key Laboratory for Biotechnology on Medicinal Plants of Jiangsu Province, School of Life Science, Jiangsu Normal University, No. 101, Shanghai Road, Tongshan District, Xuzhou, 221116 Jiangsu Province People’s Republic of China; 2 College of Health Sciences, Jiangsu Normal University, No. 101, Shanghai Road, Tongshan District, Xuzhou, 221116 Jiangsu Province People’s Republic of China

**Keywords:** CREB1, PKA, CREB, Signaling pathway, Vascular dementia, Cognitive dysfunction

## Abstract

**Background:**

As a form of dementia primarily affecting the elderly, vascular dementia (VD) is characterized by changes in the supply of blood to the brain, resulting in cognitive impairment. The aim of the present study was to explore the effects involved with cyclic adenosine monophosphate (cAMP) response element-binding (CREB)1 gene silencing on cognitive dysfunction through meditation of the protein kinase A (PKA)-CREB signaling pathway in mice with VD.

**Methods:**

Both the Morris water maze test and the step down test were applied to assess the cognitive function of the mice with VD. Immunohistochemical and TUNEL staining techniques were employed to evaluate the positive expression rates of the protein CREB1 and Cleaved Caspase-3, as well as neuronal apoptosis among hippocampal tissues in a respective manner. Flow cytometry was applied to determine the proliferation index and apoptosis rate of the hippocampal cells among each group. Reverse transcription quantitative polymerase chain reaction and Western blot analysis methods were applied to detect the expressions of cAMP, PKA and CREB in hippocampal cells.

**Results:**

Compared with the normal group, all the other groups exhibited impaired cognitive function, reduced cell numbers in the CAI area, positive expressions of CREB1 as well as positive optical density (OD) values. Furthermore, increased Cleaved Caspase-3 positive expression, OD value, proliferation index, apoptosis rate of hippocampal cells and neurons, were observed in the other groups when compared with the normal group, as well as lower expressions of cAMP, PKA and CREB1 and p-CREB1 (the shCREB1–1, H89 and shCREB1–1 + H89 groups < the VD group).

**Conclusion:**

The key findings of the present study demonstrated that CREB1 gene silencing results in aggravated VD that occurs as a result of inhibiting the PKA-CREB signaling pathway, thus exasperating cognitive dysfunction.

RETRACTED

## Background

Representing the second leading cause of senile dementia behind that of Alzheimer’s disease (AD), vascular dementia (VD) accounts for 17.6% of all cases of dementia in western countries, while studies have indicated this number to be even greater in the Eastern regions of the world, including in that of the Chinese and Japanese population’s (Battistin & Cagnin, 2010). Cognitive dysfunction is widely thought to be the classical feature exhibited by patients suffering from dementia (McGirr et al., 2016). In generally terms, VD, can be understood as an acquired intellectual damage syndrome, characterized by various cerebral vascular diseases however, is predominately associated with ischemic cerebrovascular disease (You et al., 2017). Dementia including the subtype of VD, arises from impairments in cognitive function, motor function, functional domains and memory impairments (Lee, 2011; Li et al., 2015). At present, the precise pathogenesis of VD remains largely unclear (Gong et al., 2012). Therefore, it is necessary that the finer details of the molecular mechanism underlying the condition are elucidated, in order to identify more effective future treatment approaches.

As a 43 kDa protein and transcription factor, cyclic adenosine monophosphate (cAMP) responsive element-binding proteins (CREB) are members of the bZIP transcription factor superfamily (Ramakrishnan & Pace, 2011). In addition, by performing the downstream of various signals, CREB1 possesses gene expression regulatory abilities and plays an essential role in long-term memory formation, behavioral changes, immune function, metabolic function, as well as cell survival (Sadamoto et al., 2010). A previous study demonstrated that subjects with spatial memory impairment had lower hippocampal levels of CREB1 (Brightwell et al., 2004). CREB is a member of the family of leucine-zipper transcription factors, while CREB1 has been reported to promote cell signal transduction (Li et al., 2012). What’s more, the phosphorylation of CREB1 has been highlighted due to its involvement in the synthesis of an array of proteins, of which play significant roles in neuronal functions, including that of protein kinase A (PKA) (Murphy Jr et al., 2013). PKA is the key mediator of the second messenger cAMP (Kleppe et al., 2011), and plays a positive role in the process of synaptic plasticity and long-term memory formation (Jarome et al., 2013). PKA is comprised of four sub-units: two regulatory sub-units and two catalytic sub-units, with the catalytic sub-units most commonly reported to bind to CREB as well as with the regulatory sub-units of cAMP (Hang et al., 2013). As an indispensable regulator of synaptic plasticity, the PKA/CREB signaling pathway plays a crucial role in the processes and functioning of learning and memory (Du et al., 2014). Studies have previously revealed that in the event that the PKA/CREB signaling pathway was to be inhibited, individuals would display learning and memory deficits similar to that of patients suffering from AD (Chen et al., 2012). Based on the aforementioned literature, we are of the belief that CREB1 and the PKA/CREB signaling pathway are both involved in cognitive function, including that of the processes of memory formation and behavioral changes (Zheng et al., 2016; Cheng et al., 2015). Hence, the central objective of the present study was to elucidate the relationship of the CREB1 gene, the PKA-CREB signaling pathway and VD, in an attempt to form a basis in the search for a new treatment method for patients suffering from VD.

RETRACTED

## Method

### Establishment of mouse model

A total of 80 male Kunming mice (aged 3-months), weighing approximately 34 ± 2.5 g (certificate number: 801032), were provided by the Animal Experiment Center of Hebei Medical University, and housed in controlled standard laboratory conditions (21 ± 2 °C) for one week. The rats were granted free access to food and water, placed on a 12 h light-dark cycle, with relative humidity conditions of 40% ~ 70% and noise levels < 50 dB. Ten mice were then randomly selected as the normal group, while the other 70 mice were used in order to establish the VD mouse model (Higuchi et al., 2017). The VD mouse model was established based on the following procedure: bilateral carotid artery ischemia reperfusion combined with tail bleeding, anesthetized by means of intraperitoneal injection with 40 mg/kg 0.4% pentobarbital sodium solution, and immobilized on an operating table followed by routine sterilization, and routine disinfection. Through an anterior neck middle incision, the bilateral carotid arteries were bluntly dissected. Next, a No. 4 thread buckle was hooked to the artery, and a thread was tightened in order to stop bleeding for 20 min. Meanwhile, 1 cm of the tail was cut for bleeding (0.3 ml), and the bleeding was subsequently stopped by means of heat coagulation. The next day, the conditions were observed over a period of 30 min after reperfusion, and the skin was subsequently sutured. The local skin with an incision was injected with 2000 U gentamicin. After surgery, 2000 U penicillin was intramuscularly injected at regular intervals each day for 3 consecutive days. Changes in mice physical activity post model establishment were observed in order verify as to whether successful model establishment had been obtained (De Lucia et al., 2015). The mice in the VD group exhibited behavioral changes, such as sluggishness, reduced food intake, dry hair and slow response to external stimuli. All efforts were made to minimize animal suffering.

RETRACTED

### Construction of CREB lentiviral vectors and grouping

RNA interference (RNAi) was applied to construct the shRNA lentiviral expression vector (pLenR-GPH vector) targeting CREB1 (shCREB1–1, shCREB1–2 and shCREB1–3) with the negative control (NC)-siRNA-CREB and positive control siRNA-glyceraldehyde-3-phosphate dehydrogenase (GAPDH). Based on the mRNA sequence of the NCBI nucleotide CREB1, two specific mouse CREB1 siRNA target sequences were designed. Double stranded DNA oligo comprised of interference sequences was synthesized, which were then directly connected to enzyme-digested carriers.

The mice were then assigned into 6 groups, namely: the normal, VD, NC, shCREB1 (shCREB1–1, shCREB1–2 and shCREB1–3 groups; each included 10 mice; the group exhibiting the best silence efficiency as per evaluation by means of reverse transcription quantitative polymerase chain reaction (RT-qPCR) was used for subsequent experiments), H89 (PKA-CREB signaling pathway inhibitor) and shCREB1 + H89 groups. Mice in the shCREB1 groups were injected with 20 μl of CREB1 siRNA lentiviral vectors at the caudal vein, while mice in the NC group were injected with 20 μl of unrelated sequence siRNA. An unrelated sequence of siRNA and CREB1 siRNA lentiviral vectors were encapsulated in the mixture of EntransterTM-invivo (Engreen Biosystem Co. Ltd., Beijing, China) with 10% glucose solution. Mice in the H89 group were intraperitoneal administered with 30 mg/kg 10 mol/L H89 (127243–85-0, Shanghai Peiyang Chemical Co. Ltd., Shanghai, China). The shCREB1 + H89 group were injected with CREB1 siRNA lentiviral vector, and then injected with H89. In order to ensure the identical equivalent injections were administered, all mice were injected in situ for every 72 h, with a total of three injections. After 15 d, one mouse in each of the shCREB1 groups was sacrificed by means of cervical dislocation, followed by peeling of the bilateral hippocampus. The shCREB1 group with the highest silencing efficiency was evaluated by RT-qPCR for later experiments.

### Detection of cognition function

On the 30th day, the cognition function of the mice was evaluated using the Morris water maze (MWM) test (Celik et al., 2016) and step-down test (Chi et al., 2017). In regard to the MWM test, a circular pool (130 cm in diameter and 50 cm in depth) was filled with water (19 °C–20 °C). According to the four cardinal points (at the four corners) marked in the wall, the pool was divided into four equal quadrants: the right lower, left lower, right upper and left upper. A platform was then placed in the right lower quadrant and submerged 1.5 cm below the surface of the water. (Battistin & Cagnin, 2010) The place navigation experiment was conducted according to the following: After training for 5 d, the mice were placed into the water facing the wall at the right lower, left lower, right upper and left upper quadrants successively, and the length of time required to find the platform within 2 min was recorded. The time spent finding the platform was referred to as the latent time. If the mice found the platform within 2 min, the actual latent time was then recorded, if not, it would be aided in the form of gentle guidance to the platform and stationed for 10 s, and the latent time was then recorded as 2 min. (McGirr et al., 2016) The spatial probe experiment was performed according to the following: On the sixth day, the platform was removed, in order to allow the rats to find the platform based on their memory. The swimming time was set at 120 s, and the swimming track of each mouse was recorded during the preset time of 120 s. The number of times that the original platform was crossed and the residence time at the original platform quadrant were considered to be a reflection as to whether or not the mice had remembered the location of the original platform. Data acquisition and processing was completed using the MWM automatic image acquisition system. The WX-2 mouse electro-optical stimulation conditioned reflex platform (Institute of Materia Medica, Chinese Academy of Medical Sciences, Beijing, China) was used for the step-down test. A cuboid conditioning box was employed as the platform. The mice were placed toward the wall of the pool in a successive manner. A copper grid was placed on the bottom, and 36 V of alternating current was subsequently delivered to the device. A platform, 4.5 cm in diameter and height was placed on the front left corner of the conditioning box. After 5-d of feeding, the mice were placed in a conditioning box for adaption purposes for 3 min and followed by the prompt construction of an electric circuit. The time that the mice took to jump up onto the platform and steadied themselves 5 s after electric stimulation was recorded. The test was repeated 3 times for each mouse. The reaction time, latent time and number of errors were all kept record of.

RETRACTED

### Hematoxylin and eosin (HE) staining for testing morphological changes

On the 15th d, the mice were sacrificed by means of cervical dislocation for further experiments. In each group, 4 mice were randomly selected and their brain tissues were immediately removed. The obtained brain tissues were then fixed with 4% paraformaldehyde for 24 h, dehydrated by 80%, 90%, 100% ethanol and N-butanol, and finally soaked and embedded in a wax box with 60 °C conditions. Next, 5 μm serial sections were made. After spread out and collected at 45 °C, the sections were baked for 1 h at 60 °C and dewaxed with xylene. The sections were then stained with routine HE (Beijing Solarbio Science & Technology Co. Ltd., Beijing, China), followed by dehydration with graded ethanol, cleaned with dimethylbenzene and mounted with neutral gum. Finally, the pathological changes of the hippocampal neurons in the mice were observed under an optical microscope (XP-330, Shanghai Bing Yu Optical Instrument Co. Ltd., Shanghai, China).

### Immunohistochemical staining

Six brain tissues samples were randomly selected from each group. The streptavidin-biotin complex (SABC) method (Higuchi et al., 2017) was applied in order to evaluate the intercellular adhesion molecule-1 (ICAM-1) based on the instructions of the kit (BBSW042, Shenzhen Baoan Kang Biotechnology Co. Ltd., Shenzhen, China). The samples were then fixed with formaldehyde, embedded in paraffin, and made into 4 μm serial sections. The sections were then baked in an incubator at 60 °C for 1 h, conventionally dewaxed with xylene, dehydrated by graded ethanol and soaked in 3% H_2_O_2_ for 10 min. The sections were subsequently washed in distilled water, followed by antigen retrieval for 90 s at high pressure, and cooled at room temperature and washed with PBS. After the addition of 5% bovine serum albumin (BSA) blocking solution, the sections were incubated at 37 °C for 30 min. CREB1 rabbit anti-human (1: 100) (ab81289, Abcam Inc., Cambridge, MA, USA) was added to the sections, while Cleaved Caspase-3 (ab2302, Abcam Inc., Cambridge, MA, USA) as primary antibodies, and incubated at 4 °C overnight. The sections were then washed with PBS, added with biotin-labeled goat anti-rabbit antibody (HY90046, Shanghai Heng Yuan Biotechnology Co. Ltd., Shanghai, China) (1: 100 dilution) as second antibody, and incubated at 37 °C for 30 min. The sections were subsequently rinsed with PBS, followed by the addition of streptomycin avidin-peroxidase solution (Beijing Zhongshan Biotechnology Co. Ltd., Beijing, China), and incubated at 37 °C for 30 min. Afterward, the sections were washed with PBS, visualized with chromogen 3, 3-diaminobenzidine (DAB) (Beijing Bioss Biotechnology Co. Ltd., Beijing, China) at room temperature. The sections were then soaked in hematoxylin for 5 min, and washed with running water. After, the sections were rinsed in 1% hydrochloric acid alcohol for 4 s, allowing them to return to a blue color after 20 min of washing with running water. The criterion for judging CREB1 and Cleaved Caspase-3 positive cells was based on the observation of a brownish-yellow color exhibited by the positive cells. Using a low powered microscope, the same initially selected 5 random regions were selected, and the percentage of CREB1 and Cleaved Caspase-3 positive regions in each section was analyzed by Image J V1.8.0 software (National Institutes of Health, Bethesda, Maryland, USA). The positive expression rate = number of positive cells/total number of cells.

RETRACTED

### Flow cytometry

The mice in each group sacrificed by means of decapitation, followed by stripping of the hippocampus, and fixing with 70% ethanol. Single cell suspension was prepared by mesh rubbing. The DNA staining of the apoptotic cells was performed based on the one step insertion method with iodide propidium. Expo32ADC was used to analyze the immunofluorescence data and calculate the percentage of apoptotic cells in a respective manner. Muticycle AV analysis software was applied for DNA cell cycle fitting analysis, as well as to calculate the percentage of cell distribution in each phase of the DNA histogram. The proliferation index (PI) was used to determine cell proliferation activity.

### TUNEL staining for neuronal apoptosis in hippocampal CA1 region

A total of 100 mg of hippocampal tissues were collected from each group, which were then subjected to a paraffin-embedded process, cut into sections, dewaxed and dehydrated. The sections were then cut into coronal sections according to the stereotactic atlases of the mouse brain (Wang et al., 2016a), and then fixed with 4% paraformaldehyde for 2 h. The sections were then incubated at 4 °C overnight in 20% sucrose phosphate buffer. The next day, 20 μm transverse sections of hippocampal tissue were made by − 22 °C cutting machine, followed by TUNEL staining of 10 sections of each mouse with TUNEL solution. The TUNEL Kit utilized was purchased from Boehringer Mannheim GmbH (24 Mannheim, Germany), and TUNEL staining was performed according to the instructions. The apoptotic neuronal cells were observed using a microscope, which were noted to have dark granules. In addition, 10 high power fields of vision (× 200) were selected from each group under the guidance of an optical microscope. The apoptotic nuclei and the number of cells were counted, were calculated and used to determine the apoptotic index (AI) (AI = the number of apoptotic neurons/total number of neurons) of the CA1 area in the hippocampus of each group. The procedure was repeated three time in order to obtain the mean value.

RETRACTED

### RT-qPCR

A total of 30 mg hippocampal tissues were collected from each group, followed by the addition of 1 ml of Trizol reagent (Invitrogen, Carlsbad, CA, USA), and ground in an ice bath. Total RNA was extracted from the hippocampal tissues in accordance with the instructions of the Trizol reagents. The RNA purity and concentration were detected by means of ultraviolet spectrophotometry, and then samples with a purity of A260/A280 = 1.8–2.0 were subsequently adjusted to 1 ng/μl. Next, RNA was reverse transcribed into cDNA by PrimeScriptTM RT reagent Kit (Takara, RR047A, Beijing Think-Far Technology Co. Ltd., Beijing, China), and stored at − 80 °C for further use. The primers were designed and synthesized by Shanghai Sangon Biotech Company (Shanghai, China) (Table 1). SYBR Premix Ex TaqTM II (Takara, RR047A, Beijing Think far Technology Co., Ltd., Beijing, China) was applied for RT-qPCR purposes. The reaction system was comprised of 5.0 μl of SYBR Premix Ex Taq II, 0.4 μl of upstream and downstream primers (10 μmol/L) respectively, 1 μl of cDNA templates (50 ng), and the volume was then added to 10 μl by RNA enzyme-free water. The reaction conditions were as follows: pre-denaturation at 95 °C for 30 s; denaturation at 95 °C for 5 s, anneal at 58 °C for 30 s, and extension at 72 °C for 15 s, for 40 circles. The relative mRNA expressions were analyzed based on the 2-^ΔΔCT^ method.

**Table 1:** The primer sequences of mRNA

Gene	Amplification sequences of mRNA
cAMP	F: 5’-GCTAACCTCTACCGCCTCCT-3’
	R: 5’-GGTCACTGTCCCCATACACC-3’
PKA	F: 5’-CAGGAAAGCGCTCCAGATAC-3’
	R: 5’-AAGGGAAGGTTGGCGTTACT-3’
CREB	F: 5’-TACAGGATAGACTAGCCACTT-3′
	R: 5’-AATATGTTTTCCTATCGGGGT-3’
β-actin	F: 5’-GGGCACAGTGTGGGTGAC-3’
	R: 5’-CTGGCACCACACCTTCTAC-3’

Notes: *cAMP* cyclic adenosine monophosphate, *PKA* protein kinase A, *CREB* cyclic adenosine monophosphate responsive element-binding; *mRNA* microRNA

### Western blot analysis

The bilateral cerebral hippocampi were dissected, added with protein lysate, and centrifuged at 12000 r/min for 20 min at 4 °C. An ultraviolet spectrophotometer (Shanghai Branch 752, Shanghai Daping Instrument Co. Ltd., Shanghai, China) was employed to determine the protein concentration, and then adjusted for Western blotting purposes. The extracted protein was added to the sample buffer and boiled at 95 °C for 10 min. The amount of protein per well was 30 μg. The samples were separated by 12% sodium dodecyl sulfatepolyacrylamide gel electrophoresis (SDS-PAGE) (Beijing Cellchip Biotechnology Co. Ltd., Beijing, China) at an electrophoresis voltage from 80 V to 120 V. The extracted proteins were electro transferred into 0.45 μm polyvinylidene difluoride (PVDF) membranes (Sigma Aldrich, St Louis, MO, USA). The membranes were then incubated in a blocking solution comprised of 5% nonfat dry milk, placed at room temperature and shaken for 2 h in a continuous manner. The membranes were then added with 50–100 μl rabbit anti-mouse primary antibody (1: 200, B103, Hangzhou Kitgen Biotechnology Co. Ltd., Hangzhou, China), and incubated at 4 °C overnight. The membranes were then added with 50–100 μl goat anti-rabbit secondary antibody (1: 200, cAMP, PKA, CREB and p-CREB) (SunShineBo, SN134, NanJing SunShine Biotechnology Co. Ltd., Nanjing, China), and shaken at room temperature for 2 h. Finally, the reaction was visualized using enhanced chemiluminescence (ECL) kit (0164, Shanghai Shuojia Technology Co. Ltd., Shanghai, China), exposed and then developed (21475–466, VWR, Beijing NKO-GENE Biotechnology Co. Ltd., Beijing, China). Semi-quantitative analysis and photographic fixing were made using Image-Proplus (Media Cybernetics, Bethesda, Maryland, USA).

RETRACTED

### Statistical analysis

SPSS21.0 software (IBM, Armonk, NY, USA) was used for data analysis. Measurement data were presented as mean value ± standard deviation, while comparisons between groups were conducted using single factor analysis of variance. *p* < 0.05 was considered to be statistically significant.

## Results

### VD model is established successfully

The VD model was constructed by means of bilateral carotid artery ischemia reperfusion in combination with tail bleeding. There were distinct symptoms of nerve injury among all mice with bilateral common carotid artery ligation after operation. Compared with the normal group, the mice in the VD group exhibited notably reduced food intake, physical activity, sluggish action, dry hair and no response to external stimuli. These symptoms were noted to have improved after a period of time, while food intake and physical activity remained significantly reduced in comparison with the normal group.

### The shCREB1–1 group exhibits the optimal silence efficiency and is selected for the subsequent experiments

Three shRNA groups (shCREB1–1, shCREB1–2, shCREB1–3) targeting CREB1 were constructed in order to determine the one with the best silence efficiency for subsequent experimentation. RT-qPCR (Fig. 1) results demonstrated that compared with the NC group, the expression of CREB1 in three shRNA groups (shCREB1–1, shCREB1–2, shCREB1–3) targeting CREB1 was decreased (*p* < 0.05), however no significant difference was observed in relation to the expressions of CREB1 in the positive control group (siRNA-GAPDH) (*p* > 0.05). The shCREB1–1 group displayed significantly lower expressions of CREB1 and the optimal silence efficiency, compared with the shCREB1–2 and shCREB1–3 groups (all *p* < 0.05). Therefore, the shCREB1–1 group was selected for subsequent experimentation.

RETRACTED

**Fig. 1:** The shCREB1–1 group with best silence efficiency is selected for the subsequent experiments, Notes: ^*^, *p* < 0.05, compared with the NC-siRNA-CREB1 groups; #, *p* < 0.05, compared with the shCREB1–1 group; CREB1, cyclic adenosine monophosphate responsive element-binding protein 1; NC, negative control

### Cognitive functions of mice injected with shCREB1–1 or/and H89 are impaired

In order to observe the cognitive function of mice in each group, a platform test as well as the MWM test was performed. The results of MWM test revealed that the latent time of mice in all groups decreased gradually during the five-day training period. Compared with the normal group, the latent time was significantly increased, while the number of times across the original platform as well as the time of residence in the original platform quadrant in other groups were reduced in all the other groups (*p* < 0.05); compared with the VD group, the latent time recorded was significantly increased, while the number of times recorded across the original platform and the time of residence at the original platform quadrant were reduced in the shCREB1–1, H89 and shCREB1–1 + H89 groups (*p* < 0.05) (Fig. 2a-b-c). The step-down test revealed that when compared with the normal group, there were significantly longer reaction times, notably shorter latent times and increased number of errors among the three groups (all *p* < 0.05). When compared with the VD group, the shCREB1–1, H89 and shCREB1–1 + H89 groups all had significant longer reaction times, notably shorter latent time and increased number of errors (all *p* < 0.05). There was no significant difference detected between the VD group and the NC group (*p* > 0.05) (Fig. 2d-e).

**Fig. 2:** Cognitive functions of mice injected with shCREB1–1 or/and H89 are impaired, Notes: A, the latent time of each group of mice; B, the number of crossing the original platform in each group; C, residence time of each group in the original platform quadrant; D, reaction time and latent time histogram; E, histogram of error times; ^*^, *p* < 0.05, compared with the normal group; ^#^, *p* < 0.05, compared with the VD group; VD, vascular dementia; CREB1, cyclic adenosine monophosphate responsive element-binding protein 1

### Pathological changes of hippocampal neurons among mice injected with shCREB1–1 and H89 exhibit the most significant changes

HE staining was conducted in order to explore the effects of shCREB1–1 or/and H89 on the pathological changes of the hippocampal neurons among the mice. The results of HE staining demonstrated that in the normal group, there were a number of pyramidal cells in the hippocampal CA1 area with compact and well-distributed arrangement, clear outline, neat border, large and round nucleus, distinct nucleolus, rich chromatin and limpid cytoplasm. Mice in the VD and NC groups had fewer pyramidal cells, with loose and disordered arrangements, with smaller, more deeply stained and pyknotic nucleus, in the hippocampal CA1 area. The nucleolus was faded with an intensely eosinophilic cytoplasm. Compared with the VD group, the shCREB1–1 group had fewer pyramidal cells, with a more distinct disarranged structure in the hippocampal CA1 area. The shCREB1–1 + H89 group recorded the most severe pathological changes of the hippocampal neurons (Fig. 3).

RETRACTED

**Fig. 3:** Pathological changes of hippocampal neurons of mice injected with shCREB1–1 and H89 are most serious, Note: CREB1, cyclic adenosine monophosphate responsive element-binding protein 1

### Decreased positive expression rate of CREB1 and increased cleaved Caspase-3 in the hippocampal CA1 area of mice injected with shCREB1–1 or/and H89

Immunohistochemical staining was applied in order to elucidate the mechanism of shCREB1–1 or/and H89 on the positive expression rate of CREB1 and Cleaved Caspase-3 in the hippocampal CA1 area of mice. The immunohistochemical staining results illustrated in Fig. 4, revealed that CREB1 protein was expressed in cytoplasm, depicted by brown positive granules, while the cleaved caspase-3 positive cells presented brown granules. Compared with the normal group, all the other groups were determined to have a lower OD value of CREB1 protein and higher OD value of Cleaved Caspase-3 protein in the hippocampal CA1 area (all *p* < 0.05) while comparisons with the VD group, the shCREB1–1, H89 and shCREB1–1 + H89 groups had significantly decreased average OD value of CREB1 protein and increased OD value of Cleaved Caspase-3 protein in the hippocampal CA1 area (*p* < 0.05). No significant difference was detected in the NC group.

**Fig. 4:** Decreased positive expression rate of CREB1 and increased Cleaved Caspase-3 in the hippocampal CA1 area of mice injected with shCREB1–1 or/and H89, Notes: A, the immunohistochemical staining results of CREB1 in each group (× 200); B, the histogram of the CREB1 average OD; C, the immunohistochemical staining results of Cleaved Caspase-3 in each group (× 200); D, the histogram of the Cleaved Caspase-3 average OD; ^*^, *p* < 0.05, compared with the normal group; ^#^, *p* < 0.05, compared with the VD group; CREB1, cyclic adenosine monophosphate responsive element-binding protein 1; CA1, cornu ammonis 1; VD, vascular dementia; OD, optical density

RETRACTED

### Increased PI and AI of hippocampal cells in mice injected with shCREB1–1 or/and H89

Flow cytometry was used to detect the PI and apoptotic rate of the hippocampal cells. Compared with the normal group, hippocampal cell PI and as well as the rate of apoptosis were significantly elevated in the VD group, the shCREB1–1 group, the NC group, the H89 group and the shCREB1–1 + H89 group (*p* < 0.05). Compared with the VD group, hippocampal cell PI and apoptotic rate in the shCREB1–1 group, the H89 group and the shCREB1–1 + H89 group were increased (*p* < 0.05); while no significant difference was detected in regard to PI and the rate of apoptosis of hippocampus in the NC group (*p* > 0.05) (Fig. 5).

**Fig. 5:** Increased PI and rate of apoptosis of hippocampal cells in mice injected with shCREB1–1 or/and H89, Notes: A, the apoptotic rate of hippocampal cells of mice in each group; B, the PI of hippocampal cells of mice in each group; ^*^, *p* < 0.05, compared with the normal group; ^#^, *p* < 0.05, compared with the VD group; PI, proliferation index; VD, vascular dementia; CREB1, cyclic adenosine monophosphate responsive element-binding protein 1

### Increased neuronal apoptosis in hippocampal CA1 area of mice injected with shCREB1–1 or/and H89

TUNEL staining was applied in order to detect the AI of neurons in CA1 region in the hippocampus of mice. TUNEL staining (Fig. 6) results indicated that the apoptotic granules were brown in color. When compared with the normal group, all the other groups had significantly increased AI in the hippocampal CA1 area (all *p* < 0.05). The shCREB1–1, H89 and shCREB1–1 + H89 groups had significantly increased AI in the hippocampal CA1 area when compared with the VD group (*p* < 0.05). There was no significant difference observed between the NC group and the VD group (*p* > 0.05).

**Fig. 6:** Increased neuronal apoptosis in hippocampal CA1 area of mice injected with shCREB1–1 or/and H89, Notes: A, the TUNEL staining results of CA1 in hippocampus of mice in each group (× 200); B, the histogram of apoptotic index of hippocampal CA1 neurons of mice in each group; ^*^, *p* < 0.05, compared with the normal group; ^#^, *p* < 0.05, compared with the VD group; CREB1, cyclic adenosine monophosphate responsive element-binding protein 1; VD, vascular dementia

### Decreased expression of cAMP, PKA, CREB1 and p-CREB1 in hippocampal tissues of mice with shCREB1–1 or/and H89

RT-qPCR and Western blot analysis were applied in order to identify the role of CREB1 gene silencing and PKA-CREB signaling pathway in the expression of cAMP, PKA, CREB1 and p-CREB1 in hippocampal tissues. The results (Fig. 7), of which revealed that, when compared with the normal group, all the other groups had decreased mRNA and protein expression of cAMP, PKA, CREB1 and p-CREB1 in hippocampal tissues (all *p* < 0.05). The shCREB1–1, H89 and shCREB1–1 + H89 groups had significantly decreased mRNA and protein expressions of cAMP, PKA, CREB1 and p-CREB1 in hippocampal tissues when compared with the VD group (*p* < 0.05). No significant difference was detected between the NC group and the VD group (all *p* > 0.05).

RETRACTED

**Fig. 7:** Decreased expression of cAMP, PKA, CREB1 and p-CREB1 in hippocampal tissues of mice with shCREB1–1 or/and H89, Notes: A, the histogram of the mRNA expressions of cAMP, PKA and CREB1 in hippocampal tissues of mice in each group; B, The histogram of the expressions of cAMP, PKA and CREB1 in hippocampal tissues of mice in each group; C, Gray value of cAMP, PKA and CREB1 protein bands; ^*^, *p* < 0.05, compared with the normal group; ^#^, *p* < 0.05, compared with the VD group; cAMP, cyclic adenosine monophosphate; PKA, protein kinase A; CREB1, cyclic adenosine monophosphate responsive element-binding protein 1; VD, vascular dementia

## Discussion

Patients suffering from VD are widely known to manifest motor and cognitive impairments (Li et al., 2013). Studies have shown that when compared with the general population as well as patients with AD, patients with VD exhibit lower survival rates comparatively speaking (Bruandet et al., 2009). At present, there is a scarcity of effective drugs available to treat VD (Wang, 2014). Therefore, it is extremely urgent that novel treatments are developed to provide better outcomes for patients with VD. Previous literature has, stated that CREB was involved in cognitive function (Juhasz et al., 2011). Thus the present study, set out to investigate the CREB gene, which has the potential to provide new avenues in the treatment of VD. Our study mainly demonstrated that CREB1 gene silencing aggravated cognitive dysfunction through the suppression of the PKA-CREB signaling pathway in mice with VD.

A decreased expression of CREB1, declined cognitive function, decreased hippocampal cells, and higher apoptosis was detected among the mice with VD during our study. Previous studies have revealed that patients with cognitive dysfunction resulting from AD had significantly decreased expression of CREB1, which was observed in the findings of the current study (Nagakura et al., 2013). On the basis of the results of a previously conducted study, aged-impaired rats exhibited lower expressions CREB1 when compared with normal rats (Brightwell et al., 2004). In addition, a study recently conducted showed that the degeneration of hippocampal neurons could occur as a consequence of certain types of dementias, such as AD and VD (Zarow et al., 2005), with these dementias found to share an association with the apoptosis of neuronal cells (Guo et al., 2015).

RETRACTED

Additionally, VD mice transfected with shCREB1–1 or H89 or both displayed elevated levels of cell apoptosis and decreased cell proliferation in mouse hippocampal CA1 region, as well as declined cognitive function. One study demonstrated that the degeneration of hippocampal neurons was observed among mice with disrupted CREB1 (Li et al., 2012), while a prior study highlighted the central role played by CREB1 in the development of neuronal cells in hippocampal CA1 region (Hebels et al., 2009). Evidence has been provided suggesting that increased CREB1 expression was accompanied by neuronal sprouting and increasing neurogenesis (Burcescu et al., 2005). Elisabetta Ciani et al. observed that downregulation of CREB was associated with the death of cerebellar granule neurons due to the effects of nitric oxide (Ciani et al., 2002). Importantly, studies have indicated that PKA not only activates pro-survival signals, but also acts to suppress pro-apoptotic signals induced by Rap1 (Saavedra et al., 2002). The PKA-CREB signaling pathway has also been previously emphasized upon due to its critical role in the process of memory acquisition (Vitolo et al., 2002). Interestingly, a previous study revealed that the PKA-CREB signaling pathway inhibitor could act to eliminate the beneficial effects of electroacupuncture on learning and memory (Zheng et al., 2016), which was largely consistent with the results observed in the present study, in which silencing CREB1 or inhibiting the PKA-CREB signaling pathway was suggested to promote apoptosis, aggravate cognitive dysfunction and suppress hippocampal cell proliferation.

Furthermore, hippocampal cells transfected with shCREB1–1 or H89 or shCREB1–1 + H89 had descended expression levels of cAMP, PKA, CREB1 and p-CREB1, and increased expression of Cleaved Caspase-3. It has been suggested that CREB1 is the coding gene for CREB (Serretti et al., 2011). Evidence demonstrated that CREB, which plays a significant part in nerve system (Lonze & Ginty, 2002), can be activated through the phosphorylation of serine 133 by means of activating PKA (Gao et al., 2009). Signal transduction pathways converging on CREB and the subsequent modulation of the cAMP responsive genes transcription are widely accepted to be involved in therapeutic effect (Hellmann et al., 2012). Generally, cAMP is understood to be capable of activating PKA by binding the regulatory sub-units of PKA (Etique et al., 2007). A previous study indicated that cAMP activation could be influenced by CREB and PKA (Delghandi et al., 2005). Qian-Qian Li et al. demonstrated that rats with cognitive impairment exhibited lower expression of cAMP, PKA and CREB when compared with the normal group and the acupuncture group during their study (Li et al., 2015), which was in parallels with the findings of the our study. p-CREB1 is an important transcription factor which has been reported to be implicated in fibrogenesis (Wang et al., 2016b), while lower protein levels of p-CREB in the hippocampus have been linked with memory deficit (Min et al., 2012). Cleaved caspase-3 is well known as an executioner protease of apoptosis following brain ischemia, its expression has been predominantly correlated with cellular responses to stroke such as reactive astrogliosis and the infiltration of macrophages (Wagner et al., 2011). A recent study indicated that activated caspase-3 was also found in the plaques and blood vessels in VD brains (Day et al., 2015).

RETRACTED

## Conclusion

Taken together, the present study provides encouraging evidence, illustrating that silencing of the CREB1 gene could act to exacerbate VD by inhibiting the activation of the PKA-CREB signaling pathway. Our study places emphasis on CREB1 gene and the PKA-CREB signaling pathway as a promising strategy for improved outcomes of patients with VD. Therefore, the identification of CREB1 and PKA-CREB signaling pathway may aid in facilitating the existing understanding of the mechanisms of VD, with potential of serving as a prognostic marker for the treatment of VD in the future. However, due to the limitations of sample size and fund, more detailed studies are needed to fully understand the specific mechanisms and to verify our conclusion and to explore the mechanism by which CREB1 mitigates VD in the future.
